The article "Image Video Teaching Method in College Physical Education" was retracted in 2024. Reasons: signs of a paper mill; suspected computer-generated content; unreliable results or conclusions; lack of ethics approval or compliance.

# Image Video Teaching Method in College Physical Education

**DOI:** 10.1155/2022/5277660

**Published:** 2022-08-26

**Authors:** Haibo Xu, Lun Wan

**Affiliations:** Ministry of Sports, Chongqing Jiaotong University, 400074 Chongqing, China

## Abstract

At present, traditional methods of physical education in colleges and universities are no longer able to meet the requirements of modern physical education and need to be improved. The application of the visual teaching method to the teaching of physical education in college in the classroom can best see the modern theory of physical education, which is necessary for the theory of physical education in college. On this basis, it is recommended to use the teaching method with image in the teaching of physical education in college. This document is in the form of a search query in conjunction with other search methods to perform a search. This article takes Tai Chi in the university physical education curriculum as an example. It selects two classes with no difference in number of genders and conducts traditional teaching and VR image video teaching, respectively. And from the learning situation, interest and satisfaction of the two classes analyze the degree. In this study, we found that before the experiment, the number of students with 85 scores or above in the control class was 8, accounting for 20%, 14 students with 70-85 scores, accounting for 35%, and 18 students with 60-70 scores, accounting for 45%. As could be observed, the majority of students in the control class scored between 60 and 70 points overall, with a merit rate of only 55%. In the experimental class, there are 15 students with 85 points or above, accounting for 37.5%, 18 students with 70-85 points, accounting for 45%, and 7 students with 60-70 points, accounting for 17.5%. In the experimental class, the overall score of students is between 70 and 85 points, accounting for 82.5%. The image and video teaching method can be seen to be useful in improving students' athletic achievement. In addition, the image and image instruction approach can better enhance students' interest in learning, and most students are satisfied with the image and video instruction approach.

## 1. Introduction

Traditional education is mainly centered on teachers, centered on teaching materials, focusing on standardization and ignoring innovation, and mainly on blackboard teaching, which is time-consuming, labor-intensive, small in information capacity, and relatively monotonous and rigid in information display form. With the development of current technology, it has been slowly not satisfied by students. In general, owing to the constraints of all kinds of elements, there are many drawbacks of traditional sports teaching methods in higher education, and the traditional teaching methods can not meet the needs of college sports teaching. Image video teaching is a kind of teaching method based on video images. A considerable number of colleges and universities try to apply images and videos to physical education. However, in practical application, the conditions of some colleges and universities are not perfect, and the hardware equipment can not keep up with it, which makes it impossible to apply image and video to physical education teaching. It is not widely used in physical education. Therefore, it is important to study the application of imaging pedagogy in college sport classroom teaching.

The article "Image Video Teaching Method in College Physical Education" was retracted in 2024. Reasons: signs of a paper mill; suspected computer-generated content; unreliable results or conclusions; lack of ethics approval or compliance.

The method of teaching illustrations is widely used in many studies. To explore the effect of image teaching method in the standardized training of new nurses, Kim used 43 new nurses in a control group with traditional teaching method and 50 new nurses in an observation group with image teaching method for systematic training. Then, the teaching effect of the two groups was evaluated and analyzed by the SPSS software [1, 2]. Kim's method has some reference value, but in performing its experiments, the data samples used are very small, and the result is random [3]. Saffie discussed the application effect of image video education combined with feedback in postoperative functional exercise of tibial plateau fracture. Saffie selected 60 tibial fracture patients as subjects, and 60 tibial fracture patients were classified as observation group and randomized controlled group. Among them, the control group received a standard health education model, and the observation group used a video training and feedback approach to guide physical activity based on general health education. Saffie compared the knee-length function of the two emerging teams. It was found that images and videos played an important role in fracture rehabilitation training, and the team based on the combination of video education recovered better. It has a guiding role in the degree of rehabilitation training exercise [4]. To investigate the use of participatory theory as well as video response methods in cardiopulmonary resuscitation training for advanced nursing students, Eggink et al. selected 158 volunteer graduate nurses as a research tool and randomly divided them into a control group. Among them, the experimental group used conventional teaching method and participatory teaching combined with video feedback training, while the control group only used conventional teaching method. Eggink et al. used clinical CPR attitude questionnaire and outpatient CPR willingness questionnaire to evaluate the two groups of nursing students before and after training. Eggink et al. research did not test the two groups of data, and the reliability of the experimental results was not high [5]. To explore the use of back-to-back practice combined with a video-based approach to teaching orthopedics and technology teaching, Vanikieti and Rizzo randomly divided 60 students into a test group and a control group, 30 students into each group. At the end of the teaching, questionnaire survey and unified evaluation were conducted on the two groups of interns, and the relevant results were recorded. The independent sample *t*-test and *X*^2^ test were conducted by the SPSS 23.0 software. The reliability of Vanikieti and Rizzo's research is relatively low, because other factors have not been excluded, and further improvement is needed [6].

The article "Image Video Teaching Method in College Physical Education" was retracted in 2024. Reasons: signs of a paper mill; suspected computer-generated content; unreliable results or conclusions; lack of ethics approval or compliance.

In this essay, we take Taijiquan as an example and use a combination of survey questionnaire and other study methods. In the process of questionnaire survey, we adopted the method of face-to-face distribution and face-to-face recovery, which can greatly improve the recovery rate and efficiency of the questionnaire. In addition, in this study, we selected two classes with the same number of students and no gender difference and conducted traditional teaching and video teaching, respectively. This study takes the learning situation, learning interest, and satisfaction of the two classes as the entry point for the study.

## 2. Image Video Teaching and Higher Vocational Physical Education Teaching

### 2.1. Current Situation of Physical Education in Colleges and Universities

#### 2.1.1. The Teaching Content Lacks the Pertinence of Application

In many colleges and universities, basic knowledge of physical education is limited and students' interest in sports is not high. The same teaching method leads to students' hatred of teaching physical education. And then, at present, the sports teaching of many colleges and universities lacks practical skills, the teaching of which is not shaped by the size of the students, and the teaching is not rationally selected on the basis of skill, which is also a skill, an important factor hindering the development of college physical education.

### 2.2. Physical Education Teaching Method Is Relatively Old

At present, a number of universities are championing the change of physical education teaching methods to take students into the primary role and highlight their active and proactive learning [7, 8]. However, there are still some teachers who know little about physical education teaching reform. In actual teaching, students only passively organize relevant activities. In physical education, teachers still explain sports knowledge by showing relevant sports actions and require students to practice according to demonstration actions [9, 10]. This kind of teaching method is relatively backward, which can not effectively stimulate students' enthusiasm and initiative in learning and can not make students feel the fun brought by sports, and it also has certain obstacles for students' thinking. These backward teaching methods do not play the interest, entertainment, pertinence, and professionalism of physical education, so students have no enthusiasm for sports activities, so physical education can not play a better role in supporting and consolidating professional physical fitness [11].

The article "Image Video Teaching Method in College Physical Education" was retracted in 2024. Reasons: signs of a paper mill; suspected computer-generated content; unreliable results or conclusions; lack of ethics approval or compliance.

### 2.3. Lack of Teachers

In recent years, as the number of high school candidates is increasing, colleges and universities are also expanding, so there is an increasing amount of college students and a constantly growing team of teachers, but the shortage of physical education teaching resources allocation can no longer meet the needs of physical education. Colleges and universities tend to neglect physical education and are not willing to invest more resources to expand the physical education teacher team and introduce excellent physical education teachers [12–16].

### 2.4. Image and Video Teaching

Images and videos are formed from people different forms and methods of capturing the objective world using various filming tools [17]. It can act directly or indirectly on the visual. About 75% of the information people obtain from the outside comes from the visual system, and the information obtained by the visual system mainly consists of images and videos [18, 19].

#### 2.4.1. Characteristics of Image and Video

*(1) Large Amount of Data*. Video data is usually captured by a camera or imaging device and its size depends on the performance of the device itself, such as frame rate and resolution associated with the image [20, 21]. With the advancement of modern science and technology, the production process is constantly improving, and the performance of video equipment is also improving [1, 22]. And the use of high-performance video recording and storage devices to produce video is the premise of further development of video data. The recorded video is not structured data, but audio and images are stored in the device in the form of bit data. The amount of video data is seven orders of magnitude higher than that of structured data [23, 24].

*(2) Two-Dimensional Structure*. From the perspective of features, text and image data have only spatial features; that is, the orderly distribution of characters, punctuation sets and pixel groups in space, and their structure is relatively simple. Video data is different. It has not only spatial characteristics but also temporal characteristics. The spatial feature refers to the image frame and audio state in a specific time, and the temporal feature means that the spatial state will change with time.

*(3) Rich in Content*. Video contains rich content and information, including low-level image, audio information, and high-level semantic information. Image and audio information includes image color attribute, texture attribute, audio time domain feature, frequency domain feature, acoustic perception feature, and object motion feature. The latter refers to the high-level semantics contained in the video, such as the location of the event, the person, and the description of the event process. The video contains a lot of information. The computer can only run the instructions in sequence and can not understand the high-level semantics composed of human activities from the low-level video attributes. “A thousand people read hamlets, there are a thousand hamlets”; because of different personal experience, the same video may have different semantic perception. These are the problems in video content analysis, and these must be solved. In video teaching, because everyone perceives differently, there will be ambiguity, stratification, and differentiation of understanding. Figure recognition, speech recognition, and text recognition are bridges between low-level functions and high-level video semantics.

The article "Image Video Teaching Method in College Physical Education" was retracted in 2024. Reasons: signs of a paper mill; suspected computer-generated content; unreliable results or conclusions; lack of ethics approval or compliance.

#### 2.4.2. Application of Image and Video in Physical Education Teaching

The technical level and practical application effect of image and video in sports teaching rely on the development of related science and technology. The continuous upgrading of various electronic products also has a significant impact on it. However, no matter what changes have taken place, the research on video teaching still focuses on the following three main directions:

1. Organize, collect, and produce video materials of different disciplines; focus on the key points, difficulties, and basic teaching contents of the subject; visually show them to students through video; use text to assist in explanation; and decompose the images and audio frequency of each stage for explanation
2. New teaching methods often have a variety of problems in practice, and video teaching methods also have many unexpected problems
3. Actively explore the real-time interactive teaching methods between teachers and students, use the network and other ways to transfer new knowledge and new content to students faster and more conveniently, and conduct good interactive communication with students

Due to the unique participatory and interactive nature of physical education, the teacher-student relationship has an essential role to play in teaching physical activity. A positive teacher-student rapport is more conducive to physical education. This good teacher-student relationship is slowly cultivated during teaching activities and can be achieved through more interaction among teachers and students. Traditional teaching methods focus on teachers' teaching methods and students' practice methods. The implementation of video teaching method enhances the communication and interaction among teachers and students. Further exploration and discussion in video learning can effectively improve the teacher-student relationship by strengthening the transmission and building a bridge for a good teacher-student relationship. In college physical education and the use of video teaching methods in teaching, all aspects of the requirements have been met.

The article "Image Video Teaching Method in College Physical Education" was retracted in 2024. Reasons: signs of a paper mill; suspected computer-generated content; unreliable results or conclusions; lack of ethics approval or compliance.

#### 2.4.3. Advantages of Image Video Teaching in Physical Education

The original intention of physical education teaching is to strengthen physical fitness and cultivate sentiment. Once deviated from this original intention, the quality of physical education teaching will be greatly reduced. The advantage of video image teaching is that in the process of imparting knowledge and skills, the use of image and video teaching methods can fully mobilize students' organ functions such as hearing, vision, and touch and actively participate in activities. Not only does it help to raise students' acceptance and absorption of educational information, it can also visually reproduce the difference between students' wrong behaviors and standard behaviors, thus effectively improving students' thinking ability and imagination and giving them a deeper understanding of movement process, technical structure, movement points, and movement techniques, which is of great significance to improve teaching quality. In physical education, the advantages of image video teaching are as follows:

1. Help to make up for the teacher's own shortcomings, help the teacher to explain and demonstrate the action, and highlight the key points and difficulties
2. It helps motivate students, give full play to their initiative in learning, and broaden their horizons
3. Help teachers to take the method of comparing right and wrong, and correct students' wrong actions in time
4. It can help students to establish correct visual motor imagery and effectively improve their motor skills
5. It is helpful to cultivate students' observation ability, make students set up correct sports concept, and standardize technical movements

In the conventional teaching, instructors are the major subjects of teaching, and students are the acceptors of teaching. They can only passively receive knowledge. Their motivation and initiative are limited, which is not conducive to the development of students. In multimedia network teaching, the teacher changes from a single teacher to a missionary, even with students as explorers for learning and research. Students change from passive learning to active learning. In video image teaching, students can select the content and approaches appropriate to their situation through the image and video teaching environment.

The article "Image Video Teaching Method in College Physical Education" was retracted in 2024. Reasons: signs of a paper mill; suspected computer-generated content; unreliable results or conclusions; lack of ethics approval or compliance.

Broadly speaking, it refers to all the videos used in classroom teaching activities. It can be viewed as a demonstration for students, or it can be viewed by teachers for learning analysis. In a narrow sense, video teaching is to make the knowledge, skills, and other content that teachers want to impart to students into video form, so that the teaching clip can be used by more teachers for teaching and research analysis in the future, or for teachers to analyze and reflect on their own teaching.

## 3. Research Methods and Experimental Design

### 3.1. Research Object and Experimental Design

The target of the research in this paper is college students. In this study, the physical education research was conducted with the 24-style Taijiquan in general physical education class as an example. Two classes of students were selected for the study in the laboratory. The number of students in these two classes was 40, and they were all female. There was no gender difference, so we could exclude the effect of gender difference on the results.

#### 3.1.1. Experimental Design

The experimental period was one semester. Assessment of students in both classes was conducted towards the end of the semester, and the learning status and progress of students in both classes were recorded in detail during the experiment.

### 3.2. Research Methods

#### 3.2.1. Literature Analysis

Through access to information, clear the connotation of image video teaching, access to relevant books and theoretical works, to provide a certain theoretical basis for this study.

#### 3.2.2. Logical Analysis

Through reading the relevant literature, using the knowledge of pedagogy and logic, this study collates and analyzes the experimental data and results, so as to provide the basis for the scientific and reasonable research.

#### 3.2.3. Questionnaire Survey

In the experiment, we used the method of questionnaire survey and conducted questionnaire survey before and after the experiment.

*(1) Development of Questionnaire*. The content of the questionnaire is mainly about the students' learning situation before and after the experiment. Through the investigation, we can understand the changes of college students' learning situation under the image video teaching method, including the changes of learning interest, learning achievements, and teaching method satisfaction.

*(2) Distribution and Recovery of Questionnaires*. In the process of research, we conducted a questionnaire survey. The questionnaire was distributed in the form of face-to-face distribution and face-to-face recovery, which was completed by teachers. The number of questionnaires distributed is 80. Due to the on-site collection method, a total of 80 effective surveys with 100% validity were collected. Mainly through the combination of analysis methods through the form of logic and questionnaires, statistical processing of data is carried out through statistical knowledge.

The article "Image Video Teaching Method in College Physical Education" was retracted in 2024. Reasons: signs of a paper mill; suspected computer-generated content; unreliable results or conclusions; lack of ethics approval or compliance.

### 3.3. Observation Index

#### 3.3.1. Learning Situation

In the experiment, we observed the learning situation of the two classes and analyzed the learning situation of the two classes with the completion of class hours, the standard of movement, and the overall performance evaluation as the breakthrough point.

#### 3.3.2. Interest Analysis

Before and after the experiment, questionnaire survey was conducted in two classes to analyze the change of students' interest in Taijiquan, so as to highlight the advantages of image video teaching. The calculation formula of interest degree is shown in

(1) $$\begin{array}{c} \text{Interest}=\frac{\text{Very Interested}+\text{Interested}}{\text{Very Interested}+\text{Interested}+\text{Not Interested}}\times 100\%. \end{array}$$

#### 3.3.3. Satisfaction Survey

After the experiment, a questionnaire survey was conducted in two classes to ask the students' satisfaction with the teaching methods. The calculation formula of satisfaction is shown in

(2) $$\begin{array}{c} \text{Satisfaction}=\frac{\text{Very Satisfied}+\text{Satisfied}}{\text{Very Satisfied}+\text{Satisfied}+\text{Unsatisfied}}\times 100\%. \end{array}$$

### 3.4. Data Processing

In the process of data processing, we used *t*-test between the two groups of data. If *P* < 0.05, it means that there is a difference between the two groups of data, which is statistically significant. In the test process, we need to use the *t*-test formula; the formula is shown in

(3) $$\begin{array}{c} t=\frac{{\bar{x}}_{1}-{\bar{x}}_{2}}{\sqrt{\left(S_{1}^{2}/N_{1}\right)+\left(S_{2}^{2}/N_{2}\right)}}. \end{array}$$

The mean values of the samples were as follows:

(4) $$\begin{array}{c} \bar{X}=\frac{x_{1}+x_{2}+\cdots +x_{n}}{n}. \end{array}$$

The standard deviation of the sample is as follows:

(5) $$\begin{array}{c} S=\sqrt{\frac{\sum_{i=1}^{N}{\left(x_{i}-\bar{x}\right)}^{2}}{n-1}.} \end{array}$$

The overall standard deviation was as follows:

(6) $$\begin{array}{c} S=\sqrt{\frac{\sum_{i=1}^{N}{\left(x_{i}-\bar{x}\right)}^{2}}{n}}. \end{array}$$

The article "Image Video Teaching Method in College Physical Education" was retracted in 2024. Reasons: signs of a paper mill; suspected computer-generated content; unreliable results or conclusions; lack of ethics approval or compliance.

## 4. Application Analysis of Image Video Teaching Method in Higher Vocational Physical Education Classroom Teaching

### 4.1. Analysis of Learning Situation of Students in Two Classes

The learning situation of the two classes was analyzed.

#### 4.1.1. Analysis of Class Completion

In this paper, the experimental period is one semester; the total teaching hours are 28. Then, the class completion degree of the two groups of students is analyzed, and the results are shown in Table 1 and Figure 1.

As shown in Table 1 and Figure 1, the number of students who could complete the total teaching hours in the control class was 25, or 62.5%, while the number of students in the experimental class was 38, or 95%. Therefore, the use of the image teaching method can facilitate students to complete classroom instruction.

#### 4.1.2. Comparative Analysis of Final Scores

This paper presents a comparative analysis of the final grades of the two classes in terms of both movement standards and overall performance evaluation.

*(1) Evaluation of Movement Standard*. Before and after the experiment of the two classes, the number of people whose movement standard reached above good was compared. The results are shown in Figure 2.

It can be seen from Figure 2 that before the experiment, 11 students in the control class achieved good performance or above. Therefore, there was no significant difference in the evaluation of the movement norms between the two classes before the experiment. On the other hand, after the experiment, the control class of 22 people reached good or above, accounting for 55%, while the experimental class of 36 people reached good or above; the proportion was as high as 90%. The data between the two classes had obvious differences. It can be seen that the use of image video teaching method in teaching can make students' actions more standardized.

*(2) Evaluation of Overall Performance after the Experiment*. Each exercise is divided into three grades: best, best, and average. Among them, the best score is over eighty-five, the good scores 70-85 points, and the general scores 60-70 points. The results are shown in Table 2 and Figures 3 and 4. There is also a direct relationship between the students' learning methods and their grades. The more vivid the students' learning methods are, the more impressive the students will be, and the results will also be proportional.

It can be seen from Table 2 and Figures 3 and 4 that, after the experiment, the results of the evaluation and analysis of the overall scores of the two classes were analyzed. Among them, in the control class, the number of people with 85 points or above is 8, accounting for 20%; the number of people with 70-85 points is 14, accounting for 35%; the number of people between 60 and 70 points is 18, accounting for 45%. It can be seen that in the control class, most of the students' overall scores are between 60 and 70, and the good rate is only 55%. On the other hand, in the experimental class, there are 15 students with 85 points or above, accounting for 37.5%, 18 students with 70-85 points, accounting for 45%, and 7 students with 60-70 points, accounting for 17.5%. In the experimental class, the overall score of students is between 70 and 85, with a good score of 82.5%. Therefore, the image video teaching method can effectively improve the students' sports performance.

The article "Image Video Teaching Method in College Physical Education" was retracted in 2024. Reasons: signs of a paper mill; suspected computer-generated content; unreliable results or conclusions; lack of ethics approval or compliance.

### 4.2. Analysis of Interest Change of Two Classes

Before and after the experiment, the interest of the two classes was investigated, and the students' interest in Taijiquan was asked. In the study, the interest levels were divided into three levels: very interested, interested, and not interested. The interest changes of the two classes before and after the experiment were analyzed. The results are shown in Figure 3.

In Figure 5, we can see the change of interest in the two classes before and after the experiment. Among them, before the experiment, there were 6 people from the controlled and 5 people from the laboratory class. At the level of interest, there are 12 people in the control and 13 people in the laboratory class. At the level of disinterest, there were 22 people in both the control and experimental classes. At the end of the experiment, 8 people were very interested in Taijiquan, 15 people were interested in Taijiquan, and 15 people were not interested in Taijiquan. The rate of Taijiquan in the control group was 57.5%. After the experiment, 12 people were very interested in Taijiquan, 22 people were interested in Taijiquan, and only 6 people were not interested in Taijiquan. From a statistical point of view, before the experiment, the level of interest in Taijiquan was not significantly dissimilar between the two classes. However, after the experiment, there was a statistically significant change in the level of interest between the two courses, which was statistically significant. After analysis, we believe that the image video teaching method can greatly improve students' interest in learning, motivate them to learn, and make them fall in love with physical education.

### 4.3. Satisfaction Analysis of Two Classes

At the end of the experiment, questionnaires were administered to students in both classes to analyze the satisfaction of students in both classes. In this study, satisfaction ratings were evaluated in three tiers, i.e., very satisfied, satisfied, and dissatisfied. The results of the satisfaction evaluation of both classes are illustrated in Figure 4.

The article "Image Video Teaching Method in College Physical Education" was retracted in 2024. Reasons: signs of a paper mill; suspected computer-generated content; unreliable results or conclusions; lack of ethics approval or compliance.

As shown in Figure 6, it is evident that in the controlled group, 10 were highly satisfactory with the teaching method, 14 were satisfied with the teaching method, and 16 were not satisfied with the teaching method, resulting in a 60% satisfaction rate in the control class. It is evident that most of the pupils in the control class were not very satisfied with the teaching method. Moreover, in the experimental class, there are 14 people who are very satisfied with the teaching method, 18 people are satisfied with the teaching method, and 8 people are not satisfied, so the satisfaction of the experimental class is 80%. Statistically speaking, the data between the two classes are significantly different; that is to say, the satisfaction between the two classes is statistically significant.

In this paper, the video teaching and the traditional teaching mode are compared, mainly in terms of students' classroom completion, grades, interest in the course, and the satisfaction of the two course modes. It has increased by 32.5%, indicating that the mode of film and television teaching helps students to increase their learning time. In terms of academic performance, the number of people with good academic performance has increased by 35%, which also shows that the video teaching mode makes students more interested and helps students improve their learning effect. In terms of interest in the course, student interest, and course satisfaction, students in the video teaching mode have increased by 20%, which has been improved. It also shows that the video teaching method can make students' interest, satisfaction, and learning time; the learning effect has been improved, which is conducive to the improvement of students' academic performance.

## 5. Conclusions

The modernization of teaching methods has become an important symbol of education modernization with the continuous progress of scientific technology. Being a subject that integrates knowledge transfer, skill training, and physical exercise, physical education relies more on advanced teaching methods. Video image teaching method is a modern teaching method with wide application. The Internet provides a good information and interactive platform for teaching. Educators in the information age also need to seriously consider and explore the application of video image teaching method in teaching so that it can play a greater effect in university physical education. Therefore, this paper studies the application of image video instructional method in college sport classroom teaching.

The article "Image Video Teaching Method in College Physical Education" was retracted in 2024. Reasons: signs of a paper mill; suspected computer-generated content; unreliable results or conclusions; lack of ethics approval or compliance.

This article uses research methods such as questionnaire survey and documentary analysis to research. In the research process, we conducted a questionnaire survey, which was collected face-to-face, effectively improving the questionnaire collection and efficiency. In addition, we designed a control experiment; selected two classes of students, taking Taijiquan teaching in general physical education course as an example, the students of the two classes were given traditional teaching and video teaching, respectively, and the effects of the two teaching methods were analyzed from the learning situation, interest, and satisfaction.

This study found that compared with the traditional teaching methods, the use of image video teaching method can stimulate students' interest in learning and also has a great role in promoting the improvement of students' academic performance. On the other hand, in the satisfaction survey, we can see that the image video teaching method can make students more satisfied. Therefore, we believe that in college physical education classroom teaching, we should use more advanced image video teaching method, which can not only improve students' interest in sports and improve sports performance but also achieve the purpose of physical fitness, which can mobilize students' learning enthusiasm. What is not enough in this paper is that it does not compare the influencing factors of video teaching method and only discusses it in physical education teaching, which is relatively limited and does not explain the details of current physical education teaching but only explains part of it. However, in the current era of advanced technology, video teaching is not only used in physical education but may play a role in all aspects in the future, and this novel teaching method will gradually exert traditional teaching methods, or be combined with traditional teaching methods to form a new teaching method. A new teaching method, on the basis of the original teaching effect, performance, and other aspects, will be greatly improved.

## Figures and Tables

**Figure 1:** Analysis of class completion of two classes.

**Figure 2:** Comparison of the number of students with good technical standards in the two classes before and after the experiment.

**Figure 3:** Number of students in each grade of two classes.

**Figure 4:** The proportion of grades in two classes.

**Figure 5:** Analysis of the change of interest of two classes.

The article "Image Video Teaching Method in College Physical Education" was retracted in 2024. Reasons: signs of a paper mill; suspected computer-generated content; unreliable results or conclusions; lack of ethics approval or compliance.

**Figure 6:** Satisfaction analysis of two classes.

**Table 1:** Analysis of class completion of two classes.

Class	Course content	Teaching method	Total teaching hours	Number of students completed class
Control class	24 style Taijiquan	Traditional teaching	28	38
Experimental class	24 style Taijiquan	Image video teaching	28	25

**Table 2:** Overall performance evaluation.

Class	Excellent		Good		Commonly	
	Number of people	Proportion	Number of people	Proportion	Number of people	Proportion
Control class	8	20%	14	35%	18	45%
Experimental class	15	37.5%	18	45%	7	17.5%

## Data Availability

Data sharing is not applicable to this article as no new data were created or analyzed in this study.
